The article "Ang II-AT2R increases mesenchymal stem cell migration by signaling through the FAK and RhoA/Cdc42 pathways in vitro" was retracted in 2022. Reasons: duplicated images; original data or images not available; unreliable data.

# Ang II-AT2R increases mesenchymal stem cell migration by signaling through the FAK and RhoA/Cdc42 pathways in vitro

**DOI:** 10.1186/s13287-017-0617-z

**Published:** 2017-07-12

**Authors:** Xiu-ping Xu, Hong-li He, Shu-ling Hu, Ji-bin Han, Li-li Huang, Jing-yuan Xu, Jian-feng Xie, Ai-ran Liu, Yi Yang, Hai-bo Qiu

**Affiliations:** 1 Department of Critical Care Medicine, Nanjing Zhongda Hospital, School of Medicine, Southeast University, Nanjing, 210009 People’s Republic of China; 2 Department of Critical Care Medicine, Affiliated Hospital of University of Electronic Science and Technology of China & Sichuan Provincial People’s Hospital, Chengdu, 610072 People’s Republic of China

**Keywords:** Mesenchymal stem cells, Angiotensin II, AT1R, AT2R, Cell migration, Focal adhesion kinase, Rho GTPases, F-actin

## Abstract

**Background:**

Mesenchymal stem cells (MSCs) migrate via the bloodstream to sites of injury and are possibly attracted by inflammatory factors. As a proinflammatory mediator, angiotensin II (Ang II) reportedly enhances the migration of various cell types by signaling via the Ang II receptor in vitro. However, few studies have focused on the effects of Ang II on MSC migration and the underlying mechanisms.

**Methods:**

Human bone marrow MSCs migration was measured using wound healing and Boyden chamber migration assays after treatments with different concentrations of Ang II, an AT1R antagonist (Losartan), and/or an AT2R antagonist (PD-123319). To exclude the effect of proliferation on MSC migration, we measured MSC proliferation after stimulation with the same concentration of Ang II. Additionally, we employed the focal adhesion kinase (FAK) inhibitor PF-573228, RhoA inhibitor C3 transferase, Rac1 inhibitor NSC23766, or Cdc42 inhibitor ML141 to investigate the role of cell adhesion proteins and the Rho-GTPase protein family (RhoA, Rac1, and Cdc42) in Ang II-mediated MSC migration. Cell adhesion proteins (FAK, Talin, and Vinculin) were detected by western blot analysis. The Rho-GTPase family protein activities were assessed by G-LISA and F-actin levels, which reflect actin cytoskeletal organization, were detected by using immunofluorescence.

**Results:**

Human bone marrow MSCs constitutively expressed AT1R and AT2R. Additionally, Ang II increased MSC migration in an AT2R-dependent manner. Notably, Ang II-enhanced migration was not mediated by Ang II-mediated cell proliferation. Interestingly, Ang II-enhanced migration was mediated by FAK activation, which was critical for the formation of focal contacts, as evidenced by increased Talin and Vinculin expression. Moreover, RhoA and Cdc42 were activated by FAK to increase cytoskeletal organization, thus promoting cell contraction. Furthermore, FAK, Talin, and Vinculin activation and F-actin reorganization in response to Ang II were prevented by PD-123319 but not Losartan, indicating that FAK activation and F-actin reorganization were downstream of AT2R.

The article "Ang II-AT2R increases mesenchymal stem cell migration by signaling through the FAK and RhoA/Cdc42 pathways in vitro" was retracted in 2022. Reasons: duplicated images; original data or images not available; unreliable data.

**Conclusions:**

These data indicate that Ang II-AT2R regulates human bone marrow MSC migration by signaling through the FAK and RhoA/Cdc42 pathways. This study provides insights into the mechanisms by which MSCs home to injury sites and will enable the rational design of targeted therapies to improve MSC engraftment.

## Background

Mesenchymal stem cells (MSCs) are stem cells for the connective tissues, including bone, cartilage, adipose tissue, and the tendon, and like other adult stem cells, MSCs take part in the repair processes of many injured tissues and organs [1]. A prerequisite for these cells to participate in tissue repair is migration of injected MSCs to the damaged tissues [2]. When injected intravenously, MSCs appear to preferentially home to sites of injury [3], which has been observed in tissue injuries that occur in the bone [4], liver [5], brain [6], and heart [7]. However, mechanisms regarding how MSCs migrate into the injured tissue remain unknown.

Injured tissues and organs release various factors including chemoattractants, growth factors, and inflammatory factors, which can recruit MSCs to the injured site [8]. In addition to being a physiological mediator that restores circulatory integrity, angiotensin II (Ang II) has also been reported to be involved in key events of the inflammatory process and tissue damage [9]. Together with being a proinflammatory mediator, Ang II participates in numerous life processes, including cell proliferation, apoptosis, and migration. In particular, Ang II has been proved to be a chemoattractant that directs the migration of smooth muscle cells [10], human umbilical vein endothelial cells [11], cardiac fibroblasts [12], human breast cancer cells [13], and naive T cells [14]. Accordingly, it is assumed that Ang II might be a key inflammatory factor that mediates MSC migration to sites of injury.

Ang II transduces cell signaling upon binding to its receptors, namely angiotensin II type 1 receptor (AT1R) and angiotensin II type 2 receptor (AT2R). However, no consensus has been reached on the subtype of Ang II receptors that mediates the migration of different cell types [10, 13]. Thus, there is a need to investigate the receptor subtypes and associated signaling pathways in Ang II-induced MSC migration. Moreover, previous studies have shown that Ang II can lead to the formation of focal contacts and cell contraction [15], which are the key steps in the process of cell migration [16]. Focal adhesion kinase (FAK) [17] functions as an adaptor protein to recruit other focal contact proteins or their regulators, which affects the assembly or disassembly of focal contacts. Meanwhile, FAK influences the activity of Rho-family GTPases (RhoA, Rac, and Cdc42) [18], which involves the dynamic remodeling of the actin cytoskeleton that drives cell migration. Herein, we speculated that FAK and the Rho-family GTPases might be involved in Ang II-increased MSC migration.

The article "Ang II-AT2R increases mesenchymal stem cell migration by signaling through the FAK and RhoA/Cdc42 pathways in vitro" was retracted in 2022. Reasons: duplicated images; original data or images not available; unreliable data.

In this study, we demonstrate that Ang II-AT2R promotes MSC migration. Furthermore, we found that the FAK, RhoA, and Cdc42 signaling pathways were involved in Ang II-increased migration. In brief, Ang II-AT2R signaling through activation of the FAK and RhoA/Cdc42 pathways plays a critical role in MSC migration and may guide AT2R-targeted therapy to improve the efficiency of MSC engraftment in clinical applications.

## Methods

### Human MSC culture and stimulation

Human bone marrow MSCs were purchased from Cyagen Biosciences Inc. (Guangzhou, China). The cells were identified by detecting cell surface markers and the MSC multipotent potential for differentiation toward the adipogenic, osteogenic, and chondrogenic lineages; cells were maintained as described previously [19]. Cells were passaged every 3–4 days using 0.25% trypsin–EDTA (Gibco) when they reached approximately 80% confluence and were used for the experimental protocols between passages 5 and 10 [20].

For the Ang II treatments, MSCs were serum starved for 6–8 h, and different concentrations of Ang II were added for 24 h or as indicated in the figures. To inhibit the activities of AT1R, AT2R, FAK, RhoA, Rac1, and Cdc42, cells were pretreated with AT1R antagonist Losartan (5 μM; Sigma-Aldrich, St. Louis, MO, USA), AT2R antagonist PD-123319 (5 μM; Tocris Biosciences, Bristol, UK), FAK inhibitor PF-573228 (5 μg/ml; Tocris Biosciences), RhoA inhibitor C3 transferase (5 μg/ml; Cytoskeleton, Denver, CO, USA), Rac1 inhibitor NSC23766 (50 μM; Tocris Biosciences) [21], or Cdc42 inhibitor ML141 (5 μg/ml; Tocris Biosciences) for 30 min.

### RNA isolation and quantitative real-time RT-PCR

Cells were collected, and total RNA was extracted from cells using Trizol and quantified. Reverse transcription was performed using the HiScript Q RT SuperMix (Vazyme, Piscataway , NJ, USA) for qPCR with 500 ng of RNA according to the manufacturer’s instructions (25 °C for 10 min followed by 30 min at 42 °C and an additional 5 min at 85 °C). The qRT-PCR reactions were performed using the AceQ qPCR SYBR Green Master Mix (Vazyme, Piscataway, NJ, USA) and the StepOne Plus Real Time PCR System (Life Technologies) using the cDNA produced earlier. Relative changes in gene expression were normalized to the expression levels of GAPDH and calculated using the 2(^–△△Ct^) method. The primer sequences used for PCR amplification in our study were designed based on the sequences of the genomic clones and are presented in Table 1.

The article "Ang II-AT2R increases mesenchymal stem cell migration by signaling through the FAK and RhoA/Cdc42 pathways in vitro" was retracted in 2022. Reasons: duplicated images; original data or images not available; unreliable data.

**Table 1:** Primer sequences used for PCR amplification

Gene	Primer sequence (5′–3′)
*AGTR1* (122 bp, NM_032049.3)	Forward: GGAAACAGCTTGGTGGTGAT
	Reverse: GCCCATAGTGGCAAAGTCA
*AGTR2* (100 bp, NM_000686.4)	Forward: ACATCTTCAACCTCGCTGTG
	Reverse: ACAGGTCCAAAGAGCCAGTC
*GAPDH* (138 bp, NM_002046)	Forward: CAGGAGGCATTGCTGATGAT
	Reverse: GAAGGCTGGGGCTCATTT

The cDNA was amplified with initial incubation at 95 °C for 5 min followed by 40 cycles of 10 s at 95 °C and 30 s at 60 °C, and an additional extension step at the end of the last cycle (60 s at 60 °C and 15 s at 95 °C). The PCR-amplified products were analyzed on 2.0% agarose gels, visualized by staining with ethidium bromide, and photographed under a UV light.

### Wound-healing assay (scratch assay)

MSCs were grown on six-well plates until the cells were 70–80% confluent. After 24 h, the cells reached 100% confluence, were serum starved for 6 h and treated with 100 nM Ang II, and/or were pretreated with AT1R, AT2R, FAK, RhoA, Rac1, or Cdc42 antagonists. A wound was generated by scraping the cell monolayers with a pipette tip. A nearby reference point was generated using a needle as described previously [22]. At least five randomly chosen areas were quantified using ImageJ software (NIH, Bethesda, MD, USA). Experiments were repeated three times, and an individual photograph was chosen as a representation.

### Transwell migration assay

Modified Boyden chamber assays were conducted using Transwell polyester membrane filter inserts with 8-μm pores (Corning Inc., Corning, NY, USA) at a density of 500,000 cells/ml per Transwell (upper chamber) as described previously [22]. Different coculture conditions were used in the bottom chambers of the Transwells as indicated in the figures. After culturing for 12 h, the cells from the upper chambers of the Transwells were removed, and the migrated cells on the undersides of the membranes were stained with crystal violet (Beyotime, Haimen, China). Migratory cells were imaged and counted under a light microscope (Olympus, Tokyo, Japan).

### Cell proliferation

The proliferation of human bone marrow MSCs was analyzed by 3-(4, 5-dimethylthiazol-2-yl)-2, 5-diphenyltetrazolium (MTT; Sigma, St. Louis, MO) assay. Briefly, 3×10^3^ human BM-MSCs in 200µl DMEM/F12 supplemented with 10% FBS were plated in 96-well culture plates. Grown overnight and then replaced with serum-free DMEM/F12 for an additional 6 h, then the cells were treated with different concentration of Ang II (10^-8^, 10^-7^, 10^-6^, 10^-5^, 3×10^-5^M)for another 24h. 20µl of MTT (5 mg/ml) was added to the cells, and the plates were incubated in the CO2 incubator for 4 h. The resulting formazan was then solubilized in 150 µl of dimethyl sulfoxide (DMSO; Sigma) and quantified by measuring the absorbance value (OD, optical density) of each well at 565 nm. There were six duplicate wells in each group, and the experiment was repeated at least three times.

The article "Ang II-AT2R increases mesenchymal stem cell migration by signaling through the FAK and RhoA/Cdc42 pathways in vitro" was retracted in 2022. Reasons: duplicated images; original data or images not available; unreliable data.

### Western blot analysis

Total protein from cells was extracted using RIPA lysis buffer with 1 mmol/L phenylmethylsulfonyl fluoride (PMSF) (Beyotime, Haimen, China). The protein content of the cell lysates was determined using the BCA method, and approximately 20 μg of total protein was used for each sample. Protein samples were resolved by SDS-PAGE and electrophoretically transferred onto PVDF membranes (Millipore, Bedford, MA, USA). After being blocked in 5% milk or BSA for 2 h, the membranes were incubated with FAK, Talin, Vinculin, and β-actin primary antibodies (Cell Signaling Technology, Danvers, MA, USA) at 4 °C overnight. The primary antibodies were detected with their corresponding horseradish peroxidase-conjugated secondary antibodies (HuaAn Biotechnology, Hangzhou, China). Immunoreactive bands were obtained using a chemiluminescence imaging system (ChemiQ 4800 mini; Ouxiang, Shanghai, China).

### F-actin staining by fluorescence microscopy

Cells were grown on glass coverslips until they were approximately 50% confluent and washed with PBS at 37 °C, followed by fixation with 4% paraformaldehyde in PBS for 10 min at room temperature. Cells were then washed and permeabilized with 0.5% Triton-X in PBS for 5 min. After washing, phalloidin-conjugated rhodamine (Cytoskeleton) was added at 100 nM in 200 μl of PBS. After 30-min incubation in the dark, slides were washed and stained with ﻿4', 6-diamidino-2-phenylindole (DAPI, Beyotime, Haimen, China). After mounting with anti-fade mounting media, samples were examined with a microscope (Olympus) equipped with fluorescent illumination and a digital charge-coupled-device (CCD) camera.

### Rho GTPase activity assay

GTP-bound RhoA, Rac1, and Cdc42 were measured using corresponding G-LISA Activation Assay Kits (Cytoskeleton). After stimulation, cells were washed twice with cold PBS and lysed using the lysis buffer provided by the kits for 15 min on ice, and the lysates were centrifuged at 10,000 × *g* for 1 min at 4 °C. Supernatants were aliquoted, snap-frozen in liquid nitrogen, and stored at –80 °C, as indicated by the manufacturer’s protocol. Protein concentrations were determined, and Rho GTPase activity was assessed according to the manufacturer’s instructions.

The article "Ang II-AT2R increases mesenchymal stem cell migration by signaling through the FAK and RhoA/Cdc42 pathways in vitro" was retracted in 2022. Reasons: duplicated images; original data or images not available; unreliable data.

### Statistical analysis

All statistical analyses were performed using SPSS, version 20.0 (SPSS Inc., Chicago, IL, USA). Experiments were statistically analyzed by one-way analysis of variance (ANOVA) followed by Bonferroni’s post-hoc test. Statistical significance was determined at *p* < 0.05. Data are presented as the mean ± standard deviation (SD).

## Results

### Human bone marrow MSCs constitutively express AT1R and AT2R

Cells were harvested at confluence under normal conditions for expression analyses of AT1R and AT2R mRNA, measured by RT-PCR. Determinations were made from two identical groups of human bone marrow MSCs. The results demonstrated that cultured human bone marrow MSCs in vitro expressed both AT1R and AT2R mRNA. Moreover, the AT2R mRNA expression levels were higher than that of the AT1R mRNA (Fig. 1).

**Fig. 1:** Expression of AT1R and AT2R mRNA in human bone marrow MSCs. Representative examples of phosphor images show AT1R and AT2R receptor analysis by RT-PCR using total RNA isolated from human bone marrow MSCs. *Lanes 1 and 2*, AT1R expression in human bone marrow MSCs. *Lanes 5 and 6*, AT2R expression in human bone marrow MSCs. *GAPDH* gene used as the internal loading control (*lanes 3 and 4*). *AT1R* angiotensin II type 1 receptor, *AT2R* angiotensin II type 2 receptor

### Ang II promotes the migration of human bone marrow MSCs via AT2R

To determine the dose-dependent effects of Ang II on cell migration, MSCs were treated with concentrations of 10^–8^, 10^–7^, 10^–6^, 10^–5^, and 3 × 10^–5^ M Ang II in scratch assays and Transwell assays. Ang II-induced cell migration occurred in a dose-dependent manner, with a maximal response obtained at 10^–7^ M (100 nM) Ang II (Fig. 2). To define the roles of AT1R and AT2R in Ang II-mediated MSC migration, AT1R antagonist Losartan (5 μM) and/or AT2R antagonist PD123319 (5 μM) were added 30 min prior to the Ang II treatment. PD123319 significantly inhibited Ang II-induced migration, while Losartan had no effect (Fig. 3). The results showed that the MSC migration induced by Ang II was mainly mediated by AT2R.

**Fig. 2:** Effect of different concentrations of Ang II on migration of human bone marrow MSCs. **a** Nondirectional migration ability of human bone marrow MSCs after stimulations with different concentrations of Ang II (10^–8^, 10^–7^, 10^–6^, 10^–5^, and 3 × 10^–5^ M) examined using the scratch assay. Wound sites (areas cleared of cells in the center of the scratched area) were observed and photographed at 0 and 24 h (200×). **b** Quantitative results of wound healing. **c** Directional migration ability of human bone marrow MSCs after stimulations with the different concentrations of Ang II indicated examined using the Transwell migration assay. Migrated cells on the bottom surfaces of the Transwell inserts were stained with crystal violet and observed under a microscope (200×). **d** Quantitative results of cell migration. *n* = 3; *p < 0.05 vs normal. *Ang II* angiotensin II

**Fig. 3:** Effect of AT1R and AT2R antagonists on Ang II-mediated migration of MSCs. **a** Nondirectional migration ability of MSCs after stimulation with 100 nM Ang II following pretreatment with Losartan (5 μM) and/or PD-123319 (5 μM) examined with the scratch assay. Wound sites (areas cleared of cells in the center of the scratched area) were observed and photographed at 0 and 24 h (200×). **b** Quantitative results of wound healing. **c** Directional migration ability of MSCs after stimulation with 100 nM Ang II following pretreatment with Losartan (5 μM) and/or PD-123319 (5 μM) examined using the Transwell migration assay. Migrated cells on the bottom surfaces of the Transwell inserts were stained with crystal violet and observed under a microscope (200×). **d** Quantitative results of cell migration. Significant differences were found compared with the normal group (*n* = 3; *p < 0.05) and compared with the control group (*n* = 3; ^#^ *p* < 0.05). *Ang II* angiotensin II

To determine whether different concentrations of Ang II could influence the level of receptor expression, we measured the expression levels of AT1R and AT2R mRNA. The results showed that the AT1R and AT2R mRNA levels were increased in proportion with the concentration of Ang II. However, the AT1R mRNA level induced by Ang II was maximal at the concentration of 10^–5^ M, whereas the AT2R mRNA level was maximal at the concentration of 10^–7^ M. Thereafter, both diminished progressively to the baseline (Fig. 4).

The article "Ang II-AT2R increases mesenchymal stem cell migration by signaling through the FAK and RhoA/Cdc42 pathways in vitro" was retracted in 2022. Reasons: duplicated images; original data or images not available; unreliable data.

**Fig. 4:** Effect of different concentrations of Ang II on AT1R and AT2R mRNA expression in human bone marrow MSCs. AT1R mRNA (**a**) and AT2R mRNA (**b**) expression determined by quantitative PCR after stimulations with different concentrations of Ang II (10^–8^, 10^–7^, 10^–6^, 10^–5^, and 3 × 10^–5^ M) for 12 h. *Ang II* angiotensin II, *AT1R* angiotensin II type 1 receptor, *AT2R* angiotensin II type 2 receptor

These data confirmed that Ang II-AT2R increased MSC migration, which was consistent with the AT2R expression levels.

### Ang II-induced MSC migration is not mediated through cell proliferation

To verify whether Ang II-induced MSC migration resulted from the proliferative effects of Ang II, we performed MTT assays to measure MSC proliferation after stimulations with different concentrations of Ang II. Fig. 5 shows that Ang II had no effect on MSC proliferation, which further suggests that the Ang II-increased MSC migration was not mediated by proliferation.

**Fig. 5:** Effect of Ang II on the proliferation of MSCs. MSCs were stimulated with different concentrations of Ang II (10^–8^, 10^–7^, 10^–6^, 10^–5^, and 3 × 10^–5^ M) for 24 h. Cells cultured under normal conditions served as the baseline. The proliferation rate of MSCs following stimulation was evaluated using the MTT assay. Significant differences were found compared with the normal group (*n* = 3; *p < 0.05 vs normal). *Ang II* angiotensin II, *﻿﻿OD* optical density

### Involvement of FAK, RhoA, and Cdc42 in Ang II-enhanced migration of MSCs

Given that the activation of FAK can affect cell adhesion [17] and the activities of Rho-family GTPases (RhoA, Rac1, and Cdc42) [18] that are essential for cell migration, we investigated the effect of FAK and the Rho-family GTPases on Ang II-induced MSC migration. Migration was assessed after pretreatments with an FAK inhibitor (PF-573228), RhoA inhibitor (C3 transferase), Rac1 inhibitor (NSC23766), or Cdc42 inhibitor (ML141) in the presence of Ang II. The results showed that the FAK, RhoA, and Cdc42 inhibitors prevented Ang II-enhanced MSC migration, whereas the Rac1 inhibitor had no effect (Fig. 6).

**Fig. 6:** Roles of FAK and Rho GTPases in the migration of MSCs. **a** Nondirectional migration ability of MSCs after stimulation with Ang II and/or inhibitors of FAK and the Rho GTPases examined using the scratch assay. Wound sites (areas cleared of cells in the center of the scratched area) were observed and photographed at 0 and 24 h (200×). **b** Quantitative results of wound healing. **c** Directional migration ability of MSCs after stimulation with Ang II and/or inhibitors of FAK and the Rho GTPases examined using the Transwell migration assay. Migrated cells on the bottom surfaces of the Transwell inserts were stained with crystal violet and observed under a microscope (200×). **d** Quantitative results of cell migration. *n* = 3; *p < 0.05 vs normal, ^#^ *p* < 0.05 vs the control group. *Ang II* angiotensin II

These results demonstrated that FAK, RhoA, and Cdc42 were involved in the Ang II-enhanced MSC migration.

### FAK is critical for the formation of focal contacts by MSCs after Ang II stimulation

Studies have suggested that FAK is important for the formation of focal contacts, which mediate cell adhesion [17]; we therefore assessed the expression of the key adhesion proteins, namely Talin and Vinculin, by western blot analysis after Ang II stimulation following pretreatments with or without FAK inhibitor PF-573228. We found that Ang II increased the expression of FAK, Talin, and Vinculin, which are important proteins that form structural focal contracts (Fig. 7). However, when stimulated with Ang II and PF-573228, MSCs showed significant decreases in the expression of FAK (Fig. 7a, b), Talin (Fig. 7a, c), and Vinculin (Fig. 7a, d) compared with the Ang II group. These data suggested that FAK was critical for the formation of focal contacts in the Ang II-increased migration of MSCs.

The article "Ang II-AT2R increases mesenchymal stem cell migration by signaling through the FAK and RhoA/Cdc42 pathways in vitro" was retracted in 2022. Reasons: duplicated images; original data or images not available; unreliable data.

**Fig. 7:** FAK contributed to the formation of focal contacts in Ang II-mediated migration of MSCs. **a**–**d** Immunoblot analysis of the total cell lysates performed using antibodies against FAK, Talin, and Vinculin in MSCs pretreated with Ang II (100 nM) and/or FAK inhibitor PF-573228 (5 μg/ml). Statistically significant differences are indicated (*n* = 3; *p < 0.05 vs normal, ^#^ *p* < 0.05 vs the Ang II group). *Ang II* angiotensin II, *FAK* focal adhesion kinase

### RhoA and Cdc42 activation by FAK induces F-actin organization in MSCs after stimulation with Ang II

FAK also influences the activities of Rho-family GTPases, which participate in the dynamic remodeling of the actin cytoskeleton that drives cell migration [18]. F-actin cytoskeleton networks can regulate cellular shape changes and force the migration of MSCs [23]. Therefore, we observed the actin structure by staining cells with rhodamine phalloidin as a probe for filamentous actin after treatments with the FAK or Rho-family GTPase inhibitors. We observed that MSCs stimulated by Ang II displayed more noticeable stress fibers. Meanwhile, the FAK, RhoA, or Cdc42 inhibitor pretreatments decreased F-actin organization successfully, while the Rac1 inhibitor pretreatment did not (Fig. 8a).

**Fig. 8:** Role of FAK and Rho GTPases on F-actin organization after Ang II stimulation. **a** Immunofluorescence analysis of F-actin polymerization performed using rhodamine phalloidin (F-actin; *red–orange*). Nuclei were stained with DAPI (*blue*). An overlay of the two fluorescent signals is shown (*scale bars* = 20 μm). **b**–**d** A colorimetric ELISA-based assay was used to estimate the Rho GTPase activity levels in cell lysates. Statistically significant differences are indicated (*n* = 3; *p < 0.05 vs normal, ^#^ *p* < 0.05 vs the control group). *Ang II* angiotensin II, *OD* optical density, *DAPI* 4', 6-diamidino-2-phenylindole

To further validate the effect of FAK on the activities of the Rho-family GTPases, we detected the activities of RhoA, Rac1, and Cdc42 after PF-573228 treatment. The results indicated that FAK inhibition could significantly inhibit the activation of RhoA and Cdc42, which was consistent with actin organization (Fig. 8b).

The article "Ang II-AT2R increases mesenchymal stem cell migration by signaling through the FAK and RhoA/Cdc42 pathways in vitro" was retracted in 2022. Reasons: duplicated images; original data or images not available; unreliable data.

These results suggested that the Ang II-increased migration required FAK to activate RhoA and Cdc42, which control F-actin organization in MSCs.

### Ang II induces the expression of focal adhesion proteins and the alignment of F-actin via AT2R in MSCs

To explore whether the increased expression of focal adhesion proteins and alignment of F-actin induced by Ang II was mediated through AT2R, we measured focal adhesion protein expression after the Ang II receptor was blocked. We found that when stimulated with Ang II and PD123319, MSCs showed significant decreases in the expression of FAK (Fig. 9a, b), Talin (Fig. 9a, c), and Vinculin (Fig. 9a, d) and in the alignment of F-actin (Fig. 10) compared with the Ang II group, while Losartan had no effect. This result was consistent with the corresponding migration results, suggesting that the FAK and RhoA/Cdc42 pathways were downstream of AT2R.

**Fig. 9:** Role of Ang II receptors on the activation of focal adhesion proteins. **a**–**d** Immunoblot analysis of the total cell lysates performed with antibodies against FAK, Talin, and Vinculin in MSCs pretreated with Ang II (100 nM) and/or Losartan (5 μM) and PD-123319 (5 μM). Statistically significant differences are indicated (*n* = 3; *p < 0.05 vs normal, ^#^ *p* < 0.05 vs control). *Ang II* angiotensin II, *FAK* focal adhesion kinase

**Fig. 10:** Role of Ang II receptors on F-actin polymerization. MSCs were stimulated with 100 nM Ang II after pretreatment with Losartan and/or PD-123319. Immunofluorescence analysis was performed using rhodamine phalloidin (F-actin; *red–orange*). Nuclei were stained with DAPI (*blue*). An overlay of the two fluorescent signals is shown (*scale bars* = 20 μm). *Ang II* angiotensin II*, DAPI* 4', 6-diamidino-2-phenylindole

## Discussion

In this study, we showed that Ang II can promote the migration of MSCs in an AT2R-dependent manner. Moreover, we proved that Ang II-enhanced migration is mediated by FAK activation. On the one hand, FAK activation forms the focal contacts that enhance cell adhesion. On the other hand, RhoA and Cdc42 are activated by FAK to increase the cytoskeletal organization, thus promoting cell contraction. In addition, the formation of focal contacts and organization of the cytoskeleton are mediated through AT2R. Taken together, Ang II-AT2R mediates MSC migration through the FAK and RhoA/Cdc42 pathways in vitro ( Fig. 11).

**Fig. 11:** Schematic of Ang II-AT2R-increased MSC migration by signaling through the FAK and RhoA/Cdc42 pathways. Ang II-AT2R activates FAK, leading to the formation of focal contacts and organization of the cytoskeleton, which is mediated by RhoA and Cdc42, and increases the migration of MSCs. *Ang II* angiotensin II, *AT1R* angiotensin II type 1 receptor, *AT2R* angiotensin II type 2 receptor, *FAK* focal adhesion kinase

The utilization of MSC transplantation to enhance therapeutic effects has been reported previously [8]. However, the invasive character of local transplantation might be not feasible for widespread clinical application. Thus, a successful systemic transplantation and the migratory ability of MSCs toward sites of injury are essential for enhancing the healing process [24]. Most importantly, this process is controlled by several inflammatory factors that are released at the injured site, which promote the recruitment of MSCs [25, 26]. Undoubtedly, Ang II is involved in key events of the inflammatory process and contributes to the recruitment of inflammatory cells into the injured tissue [9]; this motivated our investigation of whether Ang II could promote the migration of MSCs. Our result demonstrated that Ang II significantly enhanced the migration of MSCs in a dose-dependent manner. This is the first time we have demonstrated that Ang II can promote the migration of human bone marrow MSCs.

The article "Ang II-AT2R increases mesenchymal stem cell migration by signaling through the FAK and RhoA/Cdc42 pathways in vitro" was retracted in 2022. Reasons: duplicated images; original data or images not available; unreliable data.

Only a few studies have shown that human MSCs express Ang II receptors. It is known that these two receptors are expressed in the monkey and human HS-5 stromal cell line at the protein level [27]. Nevertheless, AT2R mRNA was not detected in human MSCs [27]. However, our study detected not only AT1R mRNA but also AT2R mRNA in cultured human bone marrow MSCs. In accordance with our findings, human MSCs express both Ang II receptors at the mRNA level [28, 29]. We did not analyze the protein expression of AT1R and AT2R because the commercially available AT1R [30, 31] and AT2R [32] antibodies are nonspecific. Thus, the determination of mRNA expression remains the only reliable approach to date for examining AT1R and AT2R expression. However, the different AT2R gene expression patterns in human MSCs can be attributed to the different sources of the cells or cell lineages. Furthermore, after stimulation using different concentrations of Ang II, the expression of both receptors was increased to different levels, which suggests that the expression level correlates with receptor function.

Previous studies have demonstrated that Ang II stimulates cellular proliferation of different types of cells, including smooth muscle cells [33], hepatic stellate cells [34], and cardiac fibroblasts [35]. Additionally, Ang II is known to promote the proliferation of hematopoietic stem cells (HSCs) [36]. To exclude the effect of Ang II-mediated stimulation of proliferation on the migration of human bone marrow MSCs, we investigated MSC proliferation using the same concentration of Ang II and found that Ang II had no effect on cell proliferation. However, Zhang et al. [37] reported that exogenous applications of Ang II could increase mouse MSC proliferation. This discrepancy might be explained by the different species origins of the MSCs. Based on these findings, we conclude that Ang II-induced human bone marrow MSC migration is not mediated through the effects of Ang II on proliferation.

The article "Ang II-AT2R increases mesenchymal stem cell migration by signaling through the FAK and RhoA/Cdc42 pathways in vitro" was retracted in 2022. Reasons: duplicated images; original data or images not available; unreliable data.

The role of the Ang II receptors in cell migration is less clear. We found that PD123319 inhibits Ang II-induced migration of MSCs in both the scratch and Transwell culture assays. Meanwhile, the migration enhanced by Ang II is consistent with the AT2R expression. In accordance with our findings, a recent study showed that PD123319 inhibits the angiotensin-induced migration of porcine vascular smooth muscle cells [10]. In contrast, PD123319 has been shown to enhance the Ang II-induced migration of keratinocytes, suggesting an inhibitory action of AT2R in cell migration [38]. There are also several studies showing that AT2R does not contribute to the effect of Ang II on the migration of vascular smooth muscle cells [39] or monocytes [40]. Intriguingly, Zhao et al. [13] showed that Ang II plays an important role in promoting human breast cancer cell migration via AT1R. These apparent discrepancies concerning the role of Ang II receptors on migration could be attributed to cell line differences.

We next investigated potential pathways that participate in Ang II-enhanced migration. In this study, we found that Ang II enhanced the expression of FAK in human bone marrow MSCs. Moreover, blocking FAK [41] using a small molecule inhibitor, PF-573228, effectively reduced Ang II-induced MSC migration to baseline levels, thus indicating that FAK plays an important role in Ang II-induced MSC migration.

Cell adhesion and cell contraction are crucial steps in cell migration and have been reviewed recently in detail by Nitzsche et al. [24] for the mechanisms of MSC migration. FAK not only affects the assembly or disassembly of focal contacts but also influences the activity of Rho-family GTPases. The regulation of the Rho family of small GTPases, which includes RhoA, Rac1, and Cdc42, is essential for controlling the dynamics of the actin cytoskeleton and actin-associated adhesions during polarized cell migration [42]. Therefore, another important finding in our study showed that PF-573228 not only inhibits the expression of focal adhesion proteins which decrease cell adhesion but also inhibits the activity of RhoA and Cdc42, which decreases formation of the F-actin network. Furthermore, the RhoA and Cdc42 inhibitors can individually reverse the enhanced migration of MSCs that is induced by Ang II. These results suggest that Ang II enhances MSC migration by signaling through the FAK and RhoA/Cdc42 pathways. It has been shown that high targeted migration of human MSCs is associated with enhanced activation of RhoA [43], which is consistent with our results. Similarly, Cdc42 activation has also been demonstrated to enhance cell migration in human corneal endothelial cells [44]. One unanticipated finding was that Rac1 had no role in Ang II-mediated migration. The reason for this is unclear, but may have something to do with differences in cell type.

The article "Ang II-AT2R increases mesenchymal stem cell migration by signaling through the FAK and RhoA/Cdc42 pathways in vitro" was retracted in 2022. Reasons: duplicated images; original data or images not available; unreliable data.

Perhaps the most significant idea in this study is the suggestion by these findings of a novel and unique role for AT2R in mediating MSC migration in response to Ang II and the establishment of FAK and RhoA/Cdc42 as a downstream target of AT2R. However, we will need to verify the function of AT2R in MSCs using animal models in future studies. It should be noted that Ang II was shown to play a role in the osteogenesis of MSCs [29] and to enhance the paracrine production of VEGF in rat MSCs [45]. Therefore, the effect of Ang II at the same concentration on the differentiating ability and paracrine action of MSCs warrants future studies.

## Conclusions

In summary, our experiments demonstrate that Ang II-AT2R activates FAK, leading to the formation of focal contacts and RhoA/Cdc42 mediating organization of the cytoskeleton, which together increase the migration of MSCs. These findings advance our understanding of the mechanisms underlying MSC homing to injury sites and enable investigators and clinicians to directly modulate the functions of these cells with the ultimate goal of generating more potent MSCs for therapeutic applications toward human diseases.

## Abbreviations

Ang II: Angiotensin II
AT1R: Angiotensin II type 1 receptor
AT2R: Angiotensin II type 2 receptor
DMEM/F12: Dulbecco’s modified Eagle’s medium/nutrient mixture F-12
FAK: Focal adhesion kinase
FBS: Fetal bovine serum
HSC: Hematopoietic stem cell
MSC: Mesenchymal stem cell
MTT: Methyl-thiazolyl-tetrazolium
PMSF: Phenylmethylsulfonyl fluoride
RT-PCR: Reverse-transcriptase polymerase chain reaction
